# Models of α-synuclein aggregation in Parkinson’s disease

**DOI:** 10.1186/s40478-014-0176-9

**Published:** 2014-12-13

**Authors:** Rosa María Giráldez-Pérez, Mónica Antolín-Vallespín, María Dolores Muñoz, Amelia Sánchez-Capelo

**Affiliations:** CIBERNED - Ser. Neurobiología – Investigación, Hospital Universitario Ramón y Cajal – IRYCIS, Ctra. Colmenar Viejo Km 9, 28034 Madrid, Spain; Departamento Fisiología, Facultad de Farmacia, Universidad de Sevilla, Sevilla, Spain; Unidad de Neurología Experimental, Hospital Universitario Ramón y Cajal – IRYCIS, Ctra. Colmenar Viejo Km 9, 28034 Madrid, Spain

**Keywords:** α-synuclein, Parkinson’s disease, Lewy body, Animal models, Smad3, Rotenone

## Abstract

Parkinson’s disease (PD) is not only characterized by motor disturbances but also, by cognitive, sensory, psychiatric and autonomic dysfunction. It has been proposed that some of these symptoms might be related to the widespread pathology of α-synuclein (α-syn) aggregation in different nuclei of the central and peripheral nervous system. However, the pathogenic formation of α-syn aggregates in different brain areas of PD patients is poorly understood. Most experimental models of PD are valuable to assess specific aspects of its pathogenesis, such as toxin-induced dopaminergic neurodegeneration. However, new models are required that reflect the widespread and progressive formation of α-syn aggregates in different brain areas. Such α-syn aggregation is induced in only a few animal models, for example perikaryon inclusions are found in rats administered rotenone, aggregates with a neuritic morphology develop in mice overexpressing either mutated or wild-type α-syn, and in Smad3 deficient mice, aggregates form extensively in the perikaryon and neurites of specific brain nuclei. In this review we focus on α-syn aggregation in the human disorder, its genetics and the availability of experimental models. Indeed, evidences show that dopamine (DA) metabolism may be related to α-syn and its conformational plasticity, suggesting an interesting link between the two pathological hallmarks of PD: dopaminergic neurodegeneration and Lewy body (LB) formation.

## Introduction

While the first description of Parkinson’s disease (PD) may date back to ancient Indian and Chinese texts from 1000 BC, the first clear medical description of this disorder was presented by James Parkinson in 1817. Some years later, in the mid-1800s, Jean-Martin Charcot separated PD from multiple sclerosis and other disorders that are also characterized by tremor, and in 1895 Brissaud formulated the hypothesis that the substantia nigra (SN) is the main brain nucleus pathologically affected in PD [1]. Subsequently, it was Friedrich Lewy who first described the protein aggregates that form in different areas of the brain of PD patients, including the dorsal vagal nucleus, locus coeruleus and globus pallidus [2]. Not long after, Trétiakoff validated Brissaud’s hypothesis in 1919 and, by examining post-mortem tissue, he described the protein aggregates in the SN and called them Lewy bodies [3,4]. Despite this long history, even today the etiology of idiopathic PD remains unknown and given the diversity of the molecular mechanisms proposed, it has been suggested that multiple factors may cause the disease [5].

PD is the second most common neurodegenerative disorder that affects the human brain. It is primarily characterized by motor symptoms like akinesia, rigidity, resting tremor and postural instability, manifestations that are mainly derived from the progressive degeneration of dopaminergic neurons in the SN *pars compacta.* Non-motor symptoms also develop that are associated with cognitive deficits (ranging from memory impairment to dementia), emotional changes (depression, apathy and anxiety), sleep perturbations, autonomic dysfunction (bladder disturbances, orthostatic hypotension, sweating), sensory symptoms (pain, visual impairment, olfactory deficit, paresthesia, ageusia) and gastrointestinal symptoms (constipation, dribbling of saliva: [6].

Although the primary motor symptoms are shared by patients, both the full presentation of the disorder and the response to treatment are quite heterogeneous [7]. It must be borne in mind that non-dopaminergic neuronal loss is also detected in some areas of the brain, for example, that of monoaminergic cells in the locus coeruleus [8] and raphe nuclei, cholinergic cells in the nucleus basalis of Meynert [9] and in the pedunculopontine tegmental nucleus [10], as well as the loss of hypocretin cells in the hypothalamus [11]. Indeed, the other pathological changes observed are widespread, with the appearance of LB inclusions in different areas of the brain (mesostriatal system, cortex, thalamus, hypothalamus, olfactory bulb or brainstem), or alterations in the autonomic system (the spinal cord, sympathetic ganglia and myenteric plexus in the gastrointestinal tract). The widespread nature of this pathology is indicative that the disorder is not just a motor alteration but rather, a sensory, cognitive, psychiatric and autonomic disorder.

## Lewy bodies in PD

A common neuropathological feature of some neurodegenerative diseases is the presence of proteinaceous inclusion bodies caused by misfolded and intracellular aggregation of proteins in many brain regions. These abnormal protein deposits may provoke LB pathologies that involve the deposition of LBs in cell bodies, or the formation of Lewy neurites (LNs) and Papp-Lantos inclusions. While the presence of LBs is a histological hallmark of PD, they are also associated with disorders such as dementia with LBs, multiple system atrophy, Alzheimer’s disease, Down’s syndrome, neurodegeneration with brain iron accumulation type I (Hallervorden-Spatz disease), progressive autonomic failure, rapid eye movement sleep disorder, parkinsonism-dementia complex of Guam, Gaucher’s disease or Pick’s disease [12].

### LB morphology

LBs are morphologically heterogeneous, with *classic LB* arising in the brainstem as cytoplasmic inclusions of 8–30 μm in diameter, with a dense eosinophilic core and a narrow pale stained rim. On haematoxylin/eosin staining, classic LBs are observed as a spherical body with a dense core surrounded by a halo [13], whereas the *cortical LBs* present in layers V-VI of the temporal, insular and cingulate cortex have no obvious halo [14-16]. A third type of LBs are known as *pale bodies*, that are rounded, pale, eosinophilic granules which lack the eosinophilic core of classic LBs, and that are only weakly and diffusely stained with eosin. These pale bodies are thought to be precursor LBs [17]. In addition, dystrophic LNs are present in axonal processes with both thread-like and spheroid forms [13,18,19].

In dementia with LB disease, inclusions seem to be morphologically homogeneous in the neocortical and paralimbic regions of the brain. In the SN, the LBs immunolabeled with α-syn and ubiquitin fall within the spectrum from diffuse to pale bodies, and to classic LBs. Indeed, this morphological diversity in the SN may represent different stages in the formation of LBs [14].

Electron microscopy has shown that the pale rim and dense core of classic LBs correspond to zones of radially-oriented straight filaments, and zones of circular profiles, respectively. Cortical LBs and LNs also contain filaments [20,21]. Three-dimensional reconstruction from serial confocal images reflects that the LB core, immunolabeled with α-syn and ubiquitin, has a concentric layered structure, with neurofilament encircling these inner layers. Indeed, a frequent continuity between LBs and LNs has been detected, indicating that LNs may evolve into LBs [22].

### LB composition

LBs are thought to be mainly composed of α-syn [23] and the morphological characterization of LBs is mostly based on immunochemistry for α-syn, ubiquitin and neurofilament. Furthermore, the α-syn in LBs undergoes post-translational modifications, such as phosphorylation, ubiquitination and oxidative nitration [24]. However, LBs also contain many different proteins [12], such as the Leucine-rich repeat kinase 2 (LRRK2: [25], histone deacetylase 6 (HDAC6: [26] and charged multivesicular body protein 2B (CHMP2B: [27], all of which are found in the core. Indeed, LRRK2 is associated with the endoplasmic reticulum of dopaminergic neurons, HDAC6 is considered a sensor of proteasomal inhibition that plays a central role in autophagy, and CHMP2B is a component of the endosomal sorting complex involved in protein degradation. The identification of proteins present in LBs may offer molecular clues to the processes that may participate in LBs formation.

Nevertheless, the comprehensive molecular composition of LBs is still unclear, although new proteomics approaches based on mass spectrometry provide an interesting approach to discover proteins not yet described in aggregates. However, the success of such approaches will depend on the techniques used to isolate LBs. One study used cortical LB-enriched fractions derived from the LB variant of Alzheimer’s disease to identify 40 LB proteins involved in phosphorylation, ubiquitination, oxidative stress or protein trafficking [28]. Laser capture microdissection of cortical LBs from neurons located in the temporal cortex of dementia with LB disease patients, allowed 296 proteins to be detected, including the chaperone HSC71, confirming the presence of chaperone molecules in LBs [29].

### Histological localization of LBs

Studies of the topographic distribution of LBs during the course of sporadic PD has enabled a classification of the stages of disease progression to be drawn up. Neurons susceptible to contain LBs have long, thin, unmyelinated or poorly myelinated axons [30] and the parkinsonian brains analyzed can nearly all be categorized into one of six different stages, based on the location of the inclusion bodies [31]:

- Stage 1: At the earliest stage, only the dorsal motor nucleus of the vagus nerve (in the lower medulla oblongata) and the anterior olfactory nucleus are affected, suggesting that the brain pathology originates in these structures.
- Stage 2: LB inclusions appear in the raphe nuclei, magnocellular reticular nuclei and locus coeruleus.
- Stage 3: The pathology occurs in the basal portions of the midbrain and forebrain, with the SNpc, amygdala, pedunculopontine tegmental nucleus, magnocellular basal forebrain nuclei, tuberomammillary nucleus and spinal cord being affected.
- Stage 4: Cortical LBs appear in the temporal mesocortex, in the allocortical CA2 of the hippocampus and in thalamic structures.
- Stage 5: The anterior cingulate, insular and subgenual mesocortex is affected, and the neocortex appears to be affected for the first time, with LBs in high order sensory association structures and in the prefrontal neocortex. The hippocampus is clearly affected in the CA1, CA3 and entorhinal cortex.
- Stage 6: LBs are present in the primary sensory areas (the auditory field), primary motor field and premotor neocortex.

This model reflects the pathological progression in PD patients (Braak PD stage 4–6), with a caudo-rostral gradient in LB deposition from the lower brainstem to the neocortex, and with both dopaminergic and non-dopaminergic areas being affected (Table 1). Some patients do not have clinical PD symptoms, but display α-syn deposition at autopsy in areas according to Braak PD stage 1–3. They are referred to as showing incidental LB disease (iLBD), considered a prodromal state of PD [32].

**Table 1:** **Overview of LB-like formation in rodent models. Brain areas with the presence of DA receptors and LB-like and/or LN-like aggregates may suggest an interaction between the dopaminergic system and α-syn (see text)**

**Brain Nucleus**	**Braak’s stage**	**PrP-A53T-α-syn mice**		**Rotenone in rats**		**Smad3 null mice**		**DA system**
X-XII	1	+++	LB- LN					Yes
OB	1	++	LB-LN					Yes
sp5	2	++	LN			++	LN	Yes
ll	2					++	LN	Yes
Sc	2	++++	LB-LN			++	LB	Yes
RF/LC	2	+++	LB- LN			++	LN	Yes
RN	2, 3	+++	LB-LN					Yes
VTA	3	+	LB- LN			++	LN	Yes
CPu	3	++	LB- LN	+++++	LB- LN	++++	LN	Yes
SN	3	+	LB- LN	+++++	LB- LN	+++++	LN	Yes
Hp	3,4					++++	LB-LN	Yes
Th	4	+++	LB-LN					Yes
M1-M2	5,6					++++	LB-LN	Yes
Cg	5,6					+++	LN	Yes
cc-ic-cp	--					+++	LN	
Pn	--					++	LB	Yes
CB	--	++++	LB-LN			++	LN	Yes
Pir	--					+++	LN	Yes
IC	--	+++	LB-LN					
SC	--	+++	LB-LN					Yes

Besides neuronal α-syn deposition in LBs and LNs, the presence of inclusions in astrocytes has been detected by silver staining. Glial inclusions are widespread in PD, both in areas with neuronal loss and gliosis (substantia nigra, locus coeruleus and dorsal vagal nucleus), and in areas with no clear neurodegeneration or gliosis (cerebral cortex, cerebral white matter, striatum, globus pallidus, thalamus, cerebellum and spinal cord: [33]. Indeed, α-syn-immunoreactive (−ir) astrocytes adopt a topographical distribution that closely parallels that of the cortical LBs [34].

However, we should consider that this disorder has a very heterogeneous clinical manifestation [35] and as yet, there is no clear significance attributed to the presence of LBs and LNs, as direct determinants of the clinical manifestations and symptoms evident in patients with PD [36,37].

### LB genetics

It is considered that most patients with PD develop the idiopathic form of the disease as opposed to that which is genetically inherited. Although, 10-30% of PD patients report a first-degree relative with the disorder, this does not necessarily reflect genetic inheritance as it may correspond with exposure to a common environmental factor [38,39]. However, it is increasingly clear that genetic factors contribute to the pathogenesis of PD and it is currently considered a multifactorial complex disorder, caused by interactions between genetic and environmental risk factors. Alternatively, only 10% of cases develop the rarer form of PD that follows Mendelian inheritance, representing 2% of late-onset and 50% of early-onset familial PD [40,41]. Studies into these familial forms have identified several causative genes related to mitochondrial or lysosomal dysfunction, protein aggregation, the proteasome system and kinase signaling [42].

LB deposition is associated with specific mutations in some of these already known genes, including α-syn (*SNCA*: [4,43] and *LRRK2* [44,45]. Moreover, the distinction between the familial and idiopathic form of PD is currently not clear in all cases, as some evidence suggests that *SNCA* or *LRKK2* mutations also participate in the sporadic disease.

#### *SNCA*

Several dominant mutations have been described in the gene encoding α-syn, *SNCA*, with varying penetrance. In 1997, the A53T missense mutation was reported in a large Italian family associated with familial PD [4]. Subsequently, two additional missense mutations in *SNCA* were also seen to be associated to familial PD, A30P [46] and E46K [47], although these point mutations are extremely rare. Duplicate and triplicate loci of *SNCA* of different sizes (from 0.4 to 4.5 Mb) have been seen to give rise to PD, which has been related to the overexpression of the wild-type protein [43,48], influencing the age of onset and severity of the disorder [49]. Indeed, *SNCA* duplications have also been reported in apparently sporadic PD patients [50] and interestingly, patients carrying these mutations present a broad clinical phenotype, even within a given family, suggesting an influence of genetic modifiers [25,51,52]. In addition, a dinucleotide repeat polymorphism (*Rep1*) has been described in the promoter region, 10 Kb upstream of the start codon, which induces *SNCA* overexpression and that may account for increased risk in 3% of non-familiar PD [53,54]. Moreover, specific haplotypes, primarily in the 3’ UTR region, may also be associated to sporadic PD [55,56].

Although *SNCA* mutations are very rare, their identification led to the association of α-syn with LBs. This protein is predominantly localized in presynaptic nerve terminals [57,58] and missense mutations may reduce its affinity for lipids, enhancing its propensity to adopt a β-sheet conformation and promoting self-assemble into oligomers and fibril formation [59]. In this sense, the A53T mutation of *SNCA* is associated with the predominantly neuritic aggregation of α-syn in the human brain [60,61] and in a mouse model [62], as well as with severe motor impairments. Alternatively, *SNCA* overexpression may decrease the density of dopaminergic vesicles and of synaptic contacts [63]. Neuropathological diagnosis of PD requires both dopaminergic neurodegeneration in the SNpc and the presence of LBs, and as described previously, the severity of the clinical manifestation has been correlated with the broad distribution of LBs [31], which may be related to the number of alleles. Both triplication and point mutations in *SNCA* are associated with the formation of cortical and subcortical LBs, and a clinical diagnosis of PD with dementia [47,64].

The *SNCA* gene and that encoding the microtubule-associated protein tau (*MAPT*) have consistently been associated in different populations of sporadic PD [65], mainly those of European origin [66]. However, such an associated was not identified in Japanese population [67], suggesting that population-specific differences may exist in the genetics of PD.

#### Leucine-rich repeat kinase 2 (LRRK2)

Point mutations in the *LRRK2* gene are frequently associated to PD, and they are found in both late onset familial and sporadic PD. *LRRK2* mutations have the highest prevalence rate in PD patients discovered to date, having been found in 10% of cases with autosomal dominant familial PD, in 3.6% of sporadic PD cases and even in 1.8% of healthy controls [44,45,68]. The presence of mutations in healthy controls may suggest a reduced and incomplete age-dependent penetrance. However, while over 80 missense variants have been identified, only seven mutations are considered pathogenic (N1437H, R1441G/C/H, Y1699C, G2019S and I2020T), most of them lying in the C-terminal half of the protein, while two others are considered as risk factors (G2385R and R1628P: [69]. Of these, G2019S is the most frequent mutation in the Caucasian population, which explains 1% of PD cases [70]. The prevalence of this mutation is strongly influenced by ethnicity and as such, it is more frequent in patients of Southern European or North African origin, and in Ashkenazi Jews (18-40% PD cases), yet it is very rare in Asians or Northern Europeans [40,69]. The risk of PD for a person who inherits this mutation is 28% at age 59 years, 51% at 69 years and 74% at 79 years [71]. The G2019S mutation gives rise to a uniform clinical phenotype that resembles sporadic PD, both in homozygous and heterozygous carriers [71].

*LRRK2* is a gene with 51 exons and it encodes a large protein with two different enzymatic activities in the same molecule: that of a kinase and a GTPase. *LRRK2* also has multiple protein interaction domains suggesting that it may serve as a scaffold for the assembly of other proteins. The G2019S mutation affects the kinase domain of the protein, with other common mutations lying in the GTPase domain or in the protein interaction domains. The function of *LRRK2* remains largely elusive but G2019S mutations enhance its kinase activity, which may mediate neural toxicity [72]. LRRK2 is widely expressed in the healthy adult brain, mainly in the endoplasmic reticulum. Interestingly, in sporadic PD patients LRRK2 is found in the core of LBs in the SN and locus coeruleus, suggesting it may contribute to LB formation [25]. Indeed, some PD patients with *LRRK2* mutations have LB pathology [73] but this is not always the case, even within a family [40]. How *LRRK2* might participate in LB formation remains unknown, although dysfunctional autophagy has been proposed [74], as well as altered solubility and aggregation of α-syn [75].

#### Recessive mutations

Homozygous or compound heterozygous mutations in the recessive genes *Parkin*, *PINK* and *DJ-1* are associated to relatively rare forms of familial PD, and these result in early onset PD and nigral dopaminergic neuronal loss. *Parkin* mutations account for around 50% of familial juvenile and early onset PD, reaching 80% in patients with onset before the age of 20 and decreasing with increasing age at onset, becoming very rare when onset occurs after the age of 50 [42]. At least 170 mutations have been described in *Parkin*, including point mutations, exon rearrangements, “indels” and duplications. Homozygous mutations with loss-of-function predominantly induce neuronal loss in the SN and locus coeruleus, in the absence of LBs. However, compound heterozygous mutations with LB pathology have been described in a minority of patients [76]. This variability may indicate some mutation-specific effect, as it has been described loss-of-function, inactivating and activating mutations [77]. Parkin is a cytosolic E3 ubiquitin ligase that transfers ubiquitin to specific protein substrates for proteasomal and autophagic degradation. Mutations may impair Parkin activity, which might reduce the clearance and aggregation of proteins. As such, these mutations could participate in decreased α-synuclein clearance [78] or alternatively, *Parkin* mutations might decrease its solubility and lead to aggregate formation [79].

Other recessive mutations are less common, such as *PINK-1* [80] and *DJ-1* [81], producing clinical manifestations broadly similar to *Parkin* mutations and in the absence of LBs.

#### GBA mutations

Glucocerebrosidase (*GBA)* mutations were first described in Gaucher’s disease, a recessive lysosomal storage disorder that may develop into parkinsonism, and PD patients may have an increased frequency of *GBA* mutations [82]. Indeed, carriers of *GBA* mutations exhibit clinical features related to early-onset, levodopa-responsive PD, experiencing hallucinations and symptoms of cognitive decline or dementia, with the abundant presence of LBs in the neocortex [83]. *GBA* mutations in PD patients confer increased susceptibility to an earlier disease onset, to have affected relatives and to develop atypical clinical manifestations [84].

## Animal models of α-syn aggregation

Animal models are used in order to study the neurobiological basis of human disorders and to develop new treatments. When examining the validity of an animal model we can consider face validity (similarity between neurological and behavioral phenotypes seen in an animal model and the human patient), construct validity (consistent with a theoretical rational, such that the molecular and cellular changes that result from genetic manipulations should be the same as those that occur in humans), and predictive validity (i.e. it should respond to pharmacological treatment as in humans) [85,86]. Face validity is a major criterion for model evaluation. One can argue that modeling of LB deposition and dopaminergic neurodegeneration may correlate to the human pathology. However, the behavioral phenotypes differ considerably between animals such as mice and humans. Thus, face validity may prove to be an unrealistic criterion for some symptoms of the disease such as motor and cognitive deficits or emotional changes. Although some researchers advocate the primacy of one of these approaches, in practice, the validity of a model should consider all three sources of evidence [87].

Considering the histopathological hallmarks of PD, models of the disorder should address the progressive loss of dopaminergic neurons in the SNpc, reduced striatal dopamine content and altered catabolism, and it should be age dependent and with progressive alteration of the animal’s movement. Furthermore, the Braak staging scheme has strongly influenced what we think would be a good animal model for PD. Indeed, the presence of LBs and LNs, the post-translational modifications observed in the human disorder, and the composition and histological localization of LBs are all central features that an animal model of PD must address. In this review we will focus on those models related to α-syn aggregation and LB-like formation.

Classical neurotoxin-induced rodent models of PD have been studied in depth and they involve treatment with 6-hydroxydopamine (oxidative stress), MPTP, rotenone and paraquat (mitochondrial complex I inhibition), PSI and epoxomicin (proteasomal inhibition), and lipopolysaccharide (glial activation). Some of these models address the toxic insult hypothesis, whereby pesticide and herbicide use can increase the risk of PD. Most of these chemical models induce degeneration of the dopaminergic neurons in the rodent and primate SN, inducing a motor syndrome that can be modulated by anti-parkinsonian medication. Indeed, the MPTP-treated primate is still the animal model used to test drugs during their selection for clinical trials in humans [88]. These models have been useful to propose pathogenic events that occur in the disease and each mechanism (oxidative stress, mitochondrial complex I inhibition, etc.) is thought to contribute to the pathogenesis of the disorder. While all these models usually display robust nigro-striatal degeneration, the formation of LB inclusions is not a common feature. In this sense, MPTP and 6-OHDA neurotoxic models have face validity related to motor features, although construct (also known as aetiological) validity are limited [89]. Indeed, the poor predictive validity of these models seems to be related to the high failure rate of new treatments in clinical trials [90].

The discovery of mutations in patients has led to the generation of different genetic models, which may prove to be a more realistic approach to study PD. Many different species and cell models are useful for genetic manipulation, including mice, *Drosophila melanogaster* and *Caenorhabditis elegans*. In this sense, several transgenic models have been described that carry *SNCA* or *LRRK2* mutations, and while many of these develop inclusions they fail to display robust neurodegeneration. Recessive models using knockout mice of PINK-1, Parkin or DJ-1 similarly fail to exhibit a nigro-striatal pathology [88]. Animal models carrying mutations in *GBA* have recently been described in the context of PD [91-93], while other animal models focus on altering the intracellular signaling of neurotrophic factors like Smad3 or on the mechanisms of aggregation of α-syn. It should be noted that most models do not capture the main hallmarks of PD in the same animal and hence, most models are only suitable to address one particular issue. However, interesting approximations for LB-like formation have been obtained with rotenone treatment, α-syn transgenesis with either wild-type or A53T mutation and in Smad3 deficient mice. Thus, the current models do appear to be useful to asses not only motor symptoms but also aetiological and predictive validity of neuroprotective molecules that could halt the pathological progression of the disease.

### Non-human primates

MPTP (1-methyl-4-phenyl-1,2,3,6-tetrahydropyridine) is a neurotoxin used in non-human primates as the most relevant animal model of PD, given its ability to induce persistent parkinsonism in humans and on the induction of selective destruction of midbrain dopaminergic neurons [94-96]. Cardinal motor symptoms of PD are reproduced in this model, as well as other non-motor symptoms such as constipation, salivation, sleep disturbance and cognitive deficits [97]. The MPTP model has limitations as the rapid toxicity results in the acute onset of neurodegeneration and neurological symptoms. Although increased α-syn immunoreactivity (−ir) within surviving neurons is detected, MPTP-affected dopaminergic neurons do not develop LBs or LNs [98].

### Rodents

#### MPTP in mice

In mice, the MPTP model must be induced in specific strains for it to be a consistent model, such as C57 and Swiss Webster mice [99]. The loss of dopaminergic neurons depends on the administration regime (from acute to chronic), ranging from 60% to 90% [88]. Acute or sub-chronic administration does not lead to the formation of inclusions and while α-syn inclusions have been detected in the study of some chronic models, this is not always replicated. In this sense, α-syn-ir was detected in dopaminergic neurons when chronic MPTP treatment was coupled with probenecid administration to block the rapid clearance of MPTP and its derivates. On examination by electron microscopy, the neurons that accumulate α-syn appeared to contain lipid droplets or secondary lysosomes covered by proteins. Although this is quite a distinct morphology to the straight filaments detected in human LBs, it was suggested that lipofuscins may be important for the development of LBs [100,101]. When MPTP was administered continuously using an osmotic minipump, ubiquitin-ir and α-syn-ir nigral inclusions formed, although their co-localization in the same cell or aggregate was not studied. Ultrastructurally, these inclusions appeared as concentric membranes containing α-syn that was transformed into fibrillar morphology [102]. However, other studies failed to find such inclusions following acute, semi-chronic or chronic MPTP treatment with probenecid or using osmotic minipumps [103-105]. Thus, further work is required before this model can be used to study aggregate formation.

#### Rotenone in rats

Rotenone is an insecticide that accumulates in the mitochondria, inhibiting complex I and promoting oxidative stress [106], as well as inhibiting the ubiquitin-proteasome system *in vitro* [107]. While this model is one of the most promising models for PD studies, it has several drawbacks since rotenone is not a selective dopaminergic neurotoxin, it produces high rates of mortality (~30%) and there is also strong variability in neurodegeneration (only observed in 50% of rats). Interestingly, peripheral treatment with rotenone induces the formation of α-syn inclusions, with a dense core and fibrillar surrounding that resembles those observed in PD [108,109]. The aggregation of α-syn may be enhanced by neonatal lipopolysaccharide (LPS) treatment, suggesting some cooperation between perinatal inflammatory processes and exposure to this pesticide [110]. *In vitro* studies have shown that rotenone induces a conformational change in α-syn and that it accelerates the rate of fibril formation [111,112]. Indeed, like the human pathology α-syn deposits are observed in the myenteric plexus [113]. In order to avoid peripheral rotenone toxicity and hence, the high mortality rate in rats, intracerebral administration of this toxin has been used, showing significant nigro-striatal neurodegeneration but not the appearance of α-syn inclusions [114]. Indeed, variability in the results obtained following peripheral administration (subcutaneous versus intravenous infusion) has limited the use of this model as a reliable tool to study PD [115,116].

Combined administration of other herbicides and fungicides, such as paraquat and Maneb also produces a high mortality rate and modest nigro-striatal neurodegeneration without LB deposition [88].

#### Proteasome inhibitors

The discovery of mutations in *parkin* and ubiquitin carboxy terminal hydrolase-1 (*UCH-L1*) in familial PD focused attention on the ubiquitin-proteasome system, suggesting that the toxicity of α-syn was associated with misfolding of the protein, and impaired proteasomal and lysosomal degradation [117]. Indeed, the combined systemic administration of the proteasome inhibitors PSI/epoxomicin produces a loss of nigro-striatal neurons and progressive motor disabilities. Moreover, inclusion bodies were observed not only in the SN but also, in the locus coeruleus, raphe and substantia innominata [118]. However, this model has proved very difficult to reproduce and the data has not been replicated in mice, rats or primates, in which only a partial response to proteasomal inhibitors is obtained [88]. This variability frustrates the use of this model in PD research. More recently, conditional genetic deletion of a proteasomal subunit in mice that disrupts 26S proteasome degradation was shown to induce the loss of dopaminergic neurons and the appearance of inclusions in SN neurons that contain ubiquitin and α-syn. Although no biochemical studies of aggregation or double-immunolabeling have been performed to clarify the nature of these inclusions, the inclusions appear to contain mitochondria and double-membraned autophagolysomes at the ultrastructural level. However, there was no resemblance of the radially oriented, straight filaments observed in LBs [119]. Indeed, in this model the accumulation of aberrant mitochondria into inclusions seems to be independent of α-syn [120].

#### Mitochondrial dysfunction

A loss of mitochondrial complex I is observed in sporadic PD that may lead to selective dopaminergic neurodegeneration due to oxidative stress [121]. Midbrain dopaminergic neurons of PD patients and elderly humans carry high levels of somatic mtDNA mutations [122]. Indeed, neurotoxins like MPTP and rotenone inhibit this mitochondrial complex [123]. Transgenic mice overexpressing wild-type α-syn induces mitochondrial fragmentation, which may predispose to neural degeneration [124], and transgenic mice overexpressing human A53T α-syn mutation also display mitochondrial abnormalities that may explain some aspects of the aggregated α-syn toxicity [125]. Disruption of the respiratory chain has been modeled in mice by deleting the gene encoding the mitochondrial transcription factor A (TFAM) in dopaminergic neurons, thereby inhibiting the transcription of mtDNA genes. Although these mice have an interesting phenotype, with impaired motor function and neurodegeneration, α-syn is not needed to express this phenotype. Indeed, the inclusions found in dopaminergic neurons have no α-syn but rather, abnormal mitochondrial membranes [126].

#### α-syn transgenesis

Different transgenic models have been developed that overexpress wild type, A53T, A30P and truncated α-syn. However, despite initial results with mutated α-syn in rodents, they have failed to translate into truly effective transgenic models of PD [127]. Attempts to overexpress or to knock-out α-syn in rodents have produced a variety of pathological abnormalities, including aggregate formation. However, no clear loss of dopaminergic neurons is observed. On the other hand, viral transduction induces rapid neurodegeneration but it is limited to the region targeted [125]. The use of cell-type promoters, such as tyrosine hydroxylase, is a limitation to transgenic overexpression that prevents the induction of the broad brain pathology observed in humans. However, this localized overexpression of α-syn (or truncated forms) may be useful to address specific features of PD. A variety of transgenic models using different promoters that drive broad expression have induced the graded appearance of α-syn aggregations with no fibrillar morphology [125,128,129]. One particularly interesting model is the transgenic A53T α-syn under the control of the mouse prion promoter, which overexpresses the mutant protein in neurons. These mice develop progressive motor failure at 8 months of age leading to paralysis and death [62]. Inclusions have been detected in different brain areas like the SN, raphe, pons, pontine reticular nuclei, locus coeruleus and deep cerebellar nuclei. The biochemical characterization of these inclusions showed SDS-insoluble α-syn aggregation into dimers, trimers and multimers, and these LB-like inclusions have a filamentous structure like human LBs [62,130]. However, as indicated, a major drawback of this model is that no dopaminergic neurodegeneration is detected in the SN. Conversely, there is neurodegeneration in areas not affected in PD, such as among motor neurons [127,131,132].

#### LRRK2 transgenesis

LRRK2 null mice have no overt dopaminergic deficit or clear pathology in the brain, although age-dependent renal atrophy is observed that is associated with the aggregation of α-syn in renal tubules of the aged kidney [133,134]. The R1441C mutation in LRRK2 generated by a knock-in strategy in mice does not induce dopaminergic neurodegeneration but rather, DA neurotransmission and D2 receptor dysfunction. However, no obvious accumulation of α-syn is detected [135]. Mice overexpressing the G2019S mutation in LRRK2 do not reproduce any obvious gross neuropathological phenotypes nor is α-syn aggregation observed, although this LRRK2 mutation may accelerate the pathogenic phenotype of A53T α-syn mice [136-138].

#### Autophagy-lysosome system

Several studies have suggested a role for autophagy in PD. The autophagy-lysosome system is a catabolic pathway involved in protein and organelle degradation. Several types of autophagy have been described, including: microautophagy; macroautophagy, engulfing large structures; and chaperone-mediated autophagy that degrades only soluble proteins in a selective manner. Cellular homeostasis of autophagy is crucial to maintain the balance between healthy and unhealthy cells [139]. In PD and related LB diseases an accumulation of autophagosomes has been described, coupled with a reduction of lysosomal markers in nigral dopaminergic neurons, suggesting a defect in lysosome-mediated clearance of α-syn aggregates [140,141]. Indeed, α-syn is physiologically degraded by both the ubiquitin-proteasome and the autophagy-lysosome system (even by the chaperone-mediated mechanism), although the mutant forms of α-syn appear to inhibit their own degradation. Hence, these pathways would appear to participate in LB formation [142,143].

In mice, deletion of the gene essential for macroautophagy (*Atg7*) in dopaminergic neurons induces progressive moderate dopaminergic loss in the SN and striatal DA depletion at an age of 9 months, although most dopaminergic neurons are resistant to the long-term stress induced by impairing autophagy. These mice have ubiquitinated-SQSTM1 inclusions in dopaminergic neurons but no abnormal aggregation of α-syn [74]. In PD patients, the translocation to the nucleus of the TFEB transcription factor (a regulator of autophagy), is dampened in midbrain dopaminergic neurons and it co-localizes with α-syn in LBs. Using adeno-associated viral vectors to model α-syn transgenesis in rats, under the control of the synapsin-1 promoter and the WPRE enhancer, stimulation of TFEB and Beclin (an activator of autophagy) was shown to rescue nigral DA neurons from α-syn toxicity [144]. These results identify interesting new mechanisms, however no clear α-syn aggregates have yet been formed by manipulating the autophagy-lysosome system.

#### Neurotrophic factors: Smad3 deficiency

GDNF and its close relative Neurturin provide functional rescue of nigro-striatal dopaminergic neurons after 6-OHDA or MPTP treatment. These results led to clinical trials into the use of these molecules in patients with PD, although the use of exogenous GDNF in clinical trials produced inconclusive results. The neuroprotective effect of this neurotrophic factor may not be translated to the clinic as GDNF fails to protect against α-syn-induced toxicity, probably due to the blockade of GDNF signaling by α-syn [145]. Indeed, transgenesis of α-syn induced by viral overexpression in the nigro-striatum, induces dystrophic terminals in the striatum containing α-syn aggregates, which are not modified by exogenous administration of GDNF [146,147].

Recently, intracellular TGF-β1 signaling has been implicated in different pathological events related to PD in a mouse model, including LB-like formation. In humans, TGF-β1 is up-regulated in the striatum and in the ventricular cerebrospinal fluid of patients with PD [148,149]. Moreover, active TGF-β1 overexpression in the nigro-striatal system of MPTP-treated mice using adenoviral vectors produces poorer survival of dopaminergic neurons and higher levels of striatal DA depletion [150,151]. However, since the effects of TGF-β1 are dose- and context-dependent [152], its overexpression may introduce a bias in studies on animal models. Smad3 deficiency, a molecule involved in the intracellular TGF-β1 signaling cascade, provides us with a new and interesting model of PD, as it promotes selective postnatal neurodegeneration of dopaminergic midbrain neurons, strong MAO-mediated catabolism of DA in the striatum and oxidative stress, as well as dampening the trophic and astrocytic support to dopaminergic neurons. Interestingly, Smad3 deficiency induces the formation of α-syn inclusions in selected brain areas, which accumulate with age in a progressive and gene dosage dependent manner. These α-syn inclusions appear in both the perikaryon (SN and paralemniscal nucleus) and in neurites (in the motor and cingulate cortices, striatum, corpus callosum and spinal cord). Indeed, these α-syn deposits are phosphorylated at Ser^129^ and ubiquitinated, and they form a core/halo distribution that resembles the deposits observed in human LBs. In other brain areas α-syn expression is associated with an irregular morphology, increased α-syn-ir staining and neurite thickness (pontine nuclei, cerebellar white matter, cerebral peduncle, diencephalic nuclei and internal capsule). Moreover, α-syn inclusions are also detected in glial cells in the cerebellum and spinal cord. Biochemical analyses show the presence of detergent-insoluble dimers, trimers and oligomers of α-syn in the ventral midbrain, motor cortex and spinal cord [153].

There is currently increasing attention being paid to the non-motor symptoms of PD, such as cognitive impairment and behavioral disorders. The hippocampus is implicated in physiological learning and memory, as well as in the cognitive dysfunction seen in some PD patients where there is an interaction with the dopaminergic system [154]. The hippocampus of PD patients is also affected by the presence of LBs [31] and in mouse models, α-syn modulates adult neurogenesis in the dentate gyrus [155]. Indeed, the accumulation of extracellular α-syn oligomers impairs hippocampal LTP and it enhances basal synaptic transmission [156]. Both triplication and point mutations of *SNCA* are associated with cortical and subcortical LB accumulation, and such patients are clinically diagnosed as PD with dementia [47,64]. These data suggest a role for the α-syn aggregates in the cognitive impairment observed in demented PD patients. Similarly, Smad3 deficient mice have α-syn inclusions in the neuronal layers of the hippocampus. Smad3 is strongly expressed in hippocampal neurons and Smad3 deficiency induces a strong decrease in adult neurogenesis in the dentate gyrus, inducing the apoptosis of early stage and highly proliferative intermediate precursor cells (IPCs). Indeed, Smad3 deficiency abolishes the induction of LTP in the dentate gyrus but not in the CA1, highlighting the specificity of this effect. Both neurogenesis and LTP induction in the adult hippocampus are two aspects of hippocampal brain plasticity related to learning and memory that decline with age, and as a result of neurological disorders [157]. Smad3 deficiency sheds light on a new interesting pathological mechanism and provides a new model of PD to be explored in which dopaminergic dysfunction, widespread α-syn inclusions and cognitive impairment co-exist.

### Invertebrate models

Several invertebrate models have been developed that recapitulate key features of human PD. *Drosophila* models of α-syn overexpression show loss of dopaminergic neurons, locomotor dysfunction and formation of α-syn inclusions. Indeed, these inclusions are observed as a core with peripherally radiating filaments [158,159]. Despite the simplicity of the nematode model *Caenorhabditis elegans*, the presence of eight dopaminergic neurons has allowed their evaluation following parkinsonian toxic and genetic insult. Overexpression of human wild-type or mutant α-syn on *C. elegans* induces dopaminergic neurodegeneration and the formation of α-syn aggregates with fibrillar morphology [160-162]. It is interesting to note that both *Drosophila* and *C. elegans* do not express α-syn and thus, other genes like LRRK2 cannot be studied in the context of α-syn inclusion formation. These models also lack the complexity of vertebrates and hence, they are not perfect models of PD but rather, they may be useful for comprehensive genetic analysis and drug screening.

## Dopamine metabolism and α-syn

Several studies associate α-syn with the DA metabolism in the presynaptic terminals. It is known that α-syn inhibits tyrosine hydroxylase, the rate limiting enzyme of DA biosynthesis [163,164], and aromatic amino acid decarboxylase, the enzyme that converts L-Dopa to DA [165]. Indeed, deregulation of DA biosynthesis in the SN induces increased toxicity to α-syn [166].

The Smad3 deficient mouse model described earlier also associates α-syn and DA metabolism, whereby Smad3 deficiency drives α-syn overexpression and aggregation, as well as the deregulation of DA turnover by inducing MAO-dependent DA catabolism, provoking a loss of dopaminergic neurons [153]. Other mouse models, such as α-syn, parkin, DJ-1 or PINK1 null mice, also display deregulated striatal DA metabolism, release or re-uptake, although without dopaminergic neuronal loss. Increased extracellular DA, decreased DAT, increased GSH levels and differences in the catabolism of DA have all been described in Parkin deficient mice [167-169]. However, neither the number of dopaminergic neurons nor the striatal DA levels and turnover are altered in DJ-1 or PINK knock-out mice. Nevertheless, the evoked DA overflow in these mice diminishes due to increased DA uptake [170] or to the decreased quantal release of DA [171], respectively. The α-syn knock-out mice have less striatal DA, enhanced activity-dependent DA release and smaller reserve pools of synaptic vesicles [172,173], which may be due to a uninhibited DA vesicular release [174]. All these mutant mice illustrate that impaired presynaptic DA metabolism, release or re-uptake may be common to PD, although the presence of α-syn aggregates and DA neuronal loss is only detected in Smad3 deficient mice. Indeed, 3,4-dihydroxyphenylacetaldehyde (DOPAL), a MAO intermediate metabolite of DA, can induce toxic aggregation of α-synuclein [175]. These data suggest that DA metabolism and α-syn interactions may underlie the susceptibility of SN neurodegeneration in PD [176].

It was recently suggested that the spread of the pathological elements in PD, as described in the Braak stages, can occur by neuron-to-neuron transmission of aggregates to healthy cells [177,178]. In this hypothesis, preformed fibrils of α-syn enter neurons, probably by endocytosis, to recruit soluble endogenous α-syn into insoluble LB- and LN-like aggregates [179,180]. Interestingly, peripheral inoculation of α-syn fibrils by intramuscular injections can propagate the pathogenic protein to brain nuclei [181]. However, another study showed that α-syn fibrils injected into transgenic mice overexpressing α-syn mutations promotes the widespread formation of α-syn inclusions in the brain of A53T but not E46K mutant mice, nor in non-transgenic mice. The authors suggest inespecificity with neurofilament of the antibodies used and that only A53T mutant mice have the capacity to induce α-syn aggregation upon exogenous administration of α-syn [182]. This aggregate transmission may be related to the existence of extracellular forms of α-syn that are released from neurons and glia by exocytosis [183]. Indeed, extracellular α-syn may induce DA release in the striatum, establishing a new link between α-syn and DA metabolism. Furthermore, α-syn function may be related to the reorganization of plasma membrane microdomains [184].

## Conformational plasticity of α-syn

Advances in cell-free systems and model cell systems have shed light on the process of α-syn aggregation. The role proposed for α-syn is in the modulation of neurotransmitter release in the presynaptic nerve terminal, as well as influencing DA neurotransmitter biosynthesis, vesicle trafficking and exocytosis. In the cytoplasm and/or vesicle lumen, α-syn is present as an intrinsically disordered protein (IDP: i.e. a monomer that lacks a well-organized secondary structure), yet when bound to membranes it adopts several conformations, such as an extended α-helix or a broken-helix [185,186]. Indeed, despite the overwhelming evidence that α-syn is a disordered monomer in solution, two recent reports suggest that the native protein exists as a helical tetramer under physiological conditions, with reduced aggregation tendencies, and that the dissociation of the tetramer into monomeric subunits promotes toxic aggregation [187,188]. Indeed, when monomeric α-syn binds to membranes, it changes its conformation to a partially helical form [189].

Many IDPs are known to interact with a large number of proteins, serving as a nodes or hubs, in a way that IDPs undergo a disorder-to-order transition upon interaction with specific partners. More than 50 proteins have been reported to interact with α-syn, although it is unknown the proportion unfolded α-syn or that which has adopted a secondary structure as a consequence of binding within the cell [186].

The α-syn peptide has 140 amino acids, with 3 distinct regions: a N-terminal (1–60 residues) that contain four imperfect repeats of KTKEGV motifs; a NAC region (61–95 residues), with 3 additional KTKEGV repeats, and the hydrophobic and amyloidogenic NAC region; a C-terminus (96–140 residues) that is enriched in acidic and proline residues, and that facilitates interactions with different proteins [185].

The major constituent of LBs is a fibrillar form of α-syn that adopts a β-sheet structure and hence, the disordered monomer or helical tetramer is transformed into highly organized fibrils in the course of this pathology. *In vitro* studies suggest a nucleation-dependent process due to a conformational transition to anti-parallel β-sheet structures, including a committed step of α-syn dimer formation [190]. Nucleation follows a sigmoidal growth profile, with an initial lag phase where the protein changes to a partially folded intermediate to form nuclei with oligomers (Figure 1). This conformational change exposes the NAC domain that can participate in hydrophobic interactions that may initiate the aggregation process. During the growth phase, the nucleus adds monomers to form larger oligomers, polarized protofibrils and finally, fibrils. In the last steady-state phase both the fibrils and monomers appear to be in equilibrium, this model therefore reflecting the addition of monomers to existing aggregates [186,191-193]. Recently, a key conformational intermediate was characterized after oligomer formation, with the appearance of stable and compact oligomers that are more damaging to cells (Figure 1). Indeed, it seems that the assembly process can be reversed and that fibrils may disaggregate to form these stable, cytotoxic oligomers [194].

**Figure 1:** **Models of α-syn aggregation and LBs formation. A** α-Syn is present in the vesicle lumen and in the cytoplasma as an intrinsically disordered protein. α-Syn bound to membranes has distinct conformation such as an extended α-helix or a broken-helix. In the pathological context, disordered monomers may lead to oligomerization and fibril formation, following a nucleation-dependent process, in which monomers are added to existing aggregates. **B** Rotenone administration in rats, A53T α-syn transgenesis in mice and Smad3 deficient mice are interesting models to study LB formation. While A53T α-syn transgenesis and Smad3 deficiency can modulate DA metabolism, rotenone and Smad3 deficiency induce oxidative stress, mechanisms that may participate in LBs formation. Indeed, proteasome and autophagy inhibitors may impair degradation of α-syn. *LRRK2* mutations may participate in LB formation by altering autophagy and α-syn solubility.

The pathogenic aggregation of α-syn can be modulated by endogenous and exogenous factor, such as metals and pesticides, genetic mutations in *SNCA*, post-translational modifications and protein-protein interactions [186]. It is not clear how α-syn bound to membranes, such as synaptic vesicles or presynaptic plasma membrane, can aggregate. One model proposes that the broken-helix membrane bound state of α-syn releases its C-terminal region, converting the protein into a partially helical membrane bound state, which may lead to oligomerization and fibril formation. Alternatively, α-helical forms of α-syn bound to membranes may inhibit fibril formation, and membrane-bound α-syn monomers may be protected from aggregation. Indeed, oligomers have a high propensity to bind to membranes, which may promote permeabilization and disrupt cellular homeostasis [195,196]. Furthermore, α-syn localizes to the nerve terminal, where modest increments in α-syn (such as those produced by gene duplication) inhibit neurotransmitter release by reducing synaptic vesicle density and by altering vesicle reclustering after endocytosis [197].

By contrast, oligomers might be kinetically detained by interactions with small molecules, inducing secondary structures such as annular pores or spheres [198-200]. The point mutations detected in the *SNCA* gene of PD patients are also endogenous factors that could accelerate α-syn aggregation *in vitro*, with A53T and G46L forming oligomers and fibrils, and A30P forming oligomers but not fibrils [201].

### Post-translational modification of α-syn

Several post-translational modifications of α-syn may occur, such as phosphorylation, truncation, ubiquitination, nitration, sumoylation and enzymatic cross-linking. In LBs, phosphorylation at serine 129 is a common α-syn modification, although its role is unclear if we consider that overexpression of the phosphorylated serine 129 isoform in animal models does not produce toxicity [202,203]. The majority of α-syn is mono- to tri-ubiquinated [204], and while poly-ubiquitination serves as a signal for α-syn degradation by the proteasome, it does not seem to be required for α-syn fibrillation and LB formation. Nevertheless, an interplay between phosphorylation and ubiquitination may render the protein more susceptible to aggregation [205]. It is estimated that 85% of all human proteins undergo N^α^-acetylation due to the activity of N^α^-acetyltransferases, probably influencing the subcellular localization of proteins, their rate of synthesis and protein-protein interactions [206]. Tetramers of α-syn seem to be N^α^-acetylated, as is probably are the aggregated α-syn isolated from PD deposits. However, N^α^-acetylation does not seem to alter protein aggregation but more likely, lipid binding [185]. Small amounts of various C-terminal truncated forms of α-syn have been detected in LBs, which exhibit greater fibrillation capacity [204]. Furthermore, four alternatively spliced forms add another level of complexity. Compared to the canonical α-syn, the three alternative isoforms aggregate significantly less, forming shorter fibrils that are arranged in parallel or with anular structures [207].

Despite the huge amount of research into the properties of α-syn aggregation, there is still no coherent picture on the structure, dynamics, and the physiological and pathological roles of α-syn. New animal models for PD need to explore LB formation in the context of neurodegeneration and DA metabolism, such as the rotenone, α-syn transgenesis and Smad3 deficient mice, in order to clearly understand the pathological mechanism of LB formation as well as to attain effective therapies for this disease.

## Abbreviations

DA: Dopamine
IDP: Intrinsically disordered protein
LB: Lewy body
LN: Lewy neurite
PD: Parkinson’s disease
SN: Substantia nigra
α-syn: α-synuclein
